The article "Healthcare Communication Role in the Detection of Unhealthy Behavior in University Students" was retracted in 2023. Reasons: signs of a paper mill; suspected computer-generated content; unreliable results or conclusions; concerns about the data.

# Healthcare Communication Role in the Detection of Unhealthy Behavior in University Students

**DOI:** 10.1155/2021/8098963

**Published:** 2021-10-06

**Authors:** Razan Alarnous, Aida Albasalah, Samar Alshawwa

**Affiliations:** ^1^Child Development Center, King Abdullah bin Abdulaziz University Hospital, Princess Nourah bint Abdulrahman University, Riyadh, Saudi Arabia; ^2^Arabic Language Department, Arts College, Princess Nourah bint Abdulrahman University, Riyadh, Saudi Arabia; ^3^Department of Pharmaceutical Sciences, College of Pharmacy, Princess Nourah bint Abdulrahman University, Riyadh, Saudi Arabia

## Abstract

The current study aims to identify unhealthy behaviors among university students, establish means of detection of unhealthy behavior, identify obstacles to digital volunteering, and explore the relationship between volunteer preferred style of volunteering and the obstacles to volunteering. Data for the study was gathered by administering an unstructured, anonymous questionnaire to 207 female university students and staff. The survey design included questions about sociodemographic characteristics, views on different facets of volunteering, unhealthy behaviors, and correlation between volunteering and unhealthy behaviors. The results revealed unhealthy behavior detected by the respondents (51.7%). Twenty-eight (13.5%) of the 207 respondents reported using social media in detecting women with offending behavior. The value of Pearson's R is 0.245; thus, it is considered as weak or no correlation. There is hence no correlation between how respondents preferred volunteer work and the obstacle to volunteering. There is not much difference in the obstacles to volunteering faced by respondents despite their preferred style of volunteering. The findings reveal that digital volunteering effectively gains ground in detecting and managing unhealthy behaviors among university students. Much more could be achieved through digital volunteering if more awareness is created and volunteering programs are designed to be more interesting and less time-consuming to allow more students to participate.

## 1. Background

The outlook of volunteering is gradually changing in the twenty-first century in manners that bring significant problems and opportunities for managing the disaster. Particularly, shifts in the pattern of paid jobs, values and lifestyles, and the latest technology have resulted in a decrease in “conventional,” high-commitment, long-term volunteering and an increase in more vast, flexible and periodic patterns of volunteering. According to [1, 2], “the commonest sources of information about healthy behaviors for university students are the media [3, 4] and social networks.” Followed by these sources of information were the World Health Organization, television, the Ministry of Health, friends, and the Internet [1, 2]. This facet reveals the significance of the Internet in conducting campaigns on health education targeted at students of higher education [3, 5], namely the various national websites [6] and international health authorities [7]. Certified announcements published by governments [2] were also part of the chief sources of information for university students.

The article "Healthcare Communication Role in the Detection of Unhealthy Behavior in University Students" was retracted in 2023. Reasons: signs of a paper mill; suspected computer-generated content; unreliable results or conclusions; concerns about the data.

Rising adulthood as the phase of life to which students of higher education belong matches a phase of personality development and education in the corporal, mental, family, sexual, emotional, and communal domains [8]. Nevertheless, scientific evidence shows an elevated occurrence of unhealthy behaviors among students of universities [9] who tend to persevere all through life and have a significant enduring impact on their health and total well-being [10]. Furthermore, students of the university should be considered emerging advancement agents, hinged on the idea that they have advantage knowledge owing to their educational background and, as a result, possess the ability to manipulate a population's health. This can be exercised either via their personal decisions, via theoretical prospective vocations, which entail responsibilities in creating health guidelines or decision-making procedures about them [11–13]. These rising adults are liable for opening a variety of precautionary options to the public based on communication of knowledge and the implementation of preventive behaviors regarding possible communicable diseases in this respect.

Digital volunteering offers immense potentials for disaster management in the aspect of disaster announcement and challenges and risks [14, 15]. Major challenges arise from strains between the command-control tradition in emergency management and the very flat and autoorganizing character of several digital volunteering. Research points out that command-control configurations “do not easily adapt to the expanding data-generating and -seeking activities by the public” [16]. Certainly, digital volunteering forms a prospective force for decentralizing and dispensing influence within emergency management. It entails not merely a shift in technology but as well a course of quick delegation of control. With enormously few obstacles to access, several new applicants are emerging in the fields of emergency and disaster response [17].

Latest technologies have therefore opened up “virtual spaces” for volunteer activism and participation that give an authority podium for people “to make their voices heard, to coordinate activities across the globe and to mobilize public opinion” [18]. From the perspective of disaster, digital volunteers are able to generate and use the virtual spaces as podiums to manage unofficial rejoinders that may or may not be incorporated with and corresponding to the official emergency management system.

The article "Healthcare Communication Role in the Detection of Unhealthy Behavior in University Students" was retracted in 2023. Reasons: signs of a paper mill; suspected computer-generated content; unreliable results or conclusions; concerns about the data.

The enormous impact of novel communications technology is another revolution that has extensive inferences because unofficial, postdisaster volunteering comes about, and incontestably all disaster volunteering. The United Nations Volunteer program states that “technological developments are opening up spaces for people to volunteer in ways that have no parallel in history” [19]. Electronic or digital volunteering “has eliminated the need for volunteerism to be tied to definite times and locations. Thus, it greatly increases the freedom and flexibility of volunteer engagement and complements the outreach and impact of volunteers serving in situ” [19]. The burst in mobile technology and social media, in particular, has lowered the information and communication impediments to partaking in disaster response and recovery [17]. Therefore, it has facilitated development in “digitally enabled volunteering” due to disasters that occur both digitally and physically, or, as is frequently the case, in interaction [20, 21]. Meier [22] and Zook et al. [23] stated that “the trend of digital volunteering, in particular, has earned noteworthy research attention since the immense response of digital volunteers to the 2010 Haiti earthquake.” This was a turning point event that paved the way for “digital humanitarianism” that is global in reach [17]. To a large extent, online volunteers have been reported to be more successful than conventional government organizations at organizing, collating, managing, and disseminating the “data deluge” that is prompted by disasters in the Internet age in close to real-time to increase conditional awareness [24]. According to Haworth and Bruce, a key strength of digital volunteering arises from the huge capability of the Internet to facilitate crowdsourcing, mostly for volunteered geographic information (VGI). VGI “involves the sharing and mapping of spatial data through voluntary information gathered by the general public” [15], and it is especially influential for disaster circumstances. This is progressively more recognized by well-known actors. Conspicuously, the Information Services Section (ISS) of the United Nations Office for the Coordination of Humanitarian Affairs (OCHA) started a digital volunteering network—The Standby Taskforce—to create live, crowdsourced crisis maps for the 2011 Libyan revolution that was afterward used by humanitarian organizations to coordinate their relief activities [22].

The article "Healthcare Communication Role in the Detection of Unhealthy Behavior in University Students" was retracted in 2023. Reasons: signs of a paper mill; suspected computer-generated content; unreliable results or conclusions; concerns about the data.

Unhealthy behavior refers to any action an individual takes with intensity or at a rate that raises the risk of injury or disease [25]. It might sum up into a risky way of life that influences emotions, cognitive performance, and the general value of life. A great deal of the sicknesses and deaths result from individuals' behavioral styles, polluted environment, poverty, or psychological affairs [26]. A research carried out by Poortinga established that many university students binge drink, smoke tobacco, do not eat sufficient fruits and vegetables, and do not exercise enough. The study in [27] identified five groups of behaviors that have been found consistently to associate with increased sickness and death. The list includes “low levels of physical activity and high levels of sedentary activity; eating a diet high in fat and sodium, calories, and low in nutrients; smoking cigarettes; substances abuse including alcohol, illicit and remedy drugs, and risky sexual behaviors” [28]. Latest advancements in brain research have established a precarious connection between youths and unhealthy behaviors, expounding the reality that adolescence is the significant stage of risk for both unhealthy behaviors and their outcome. Adults are less susceptible to unhealthy behavior than adolescents because the sections of the brain that control decision-making, judgment, impulse control, and emotion are not yet completely developed in adolescents. Thus, teens are more likely to take risks than adults, including engaging in dangerous behaviors and experimenting with drug abuse [29]. The chances of undertaking several unhealthy behaviors increase over the process of growth, principally during the teenage years. Through sexual risk, physical risks, and experimentation with substances, some adolescents attain unhealthy behaviors and peers that endure and dampen the cultivation of other self-regulatory attitudes. Notwithstanding efforts made towards health promotion, young adults continue to practice high levels of unhealthy behaviors, as established by [30]. It is essential to understand unhealthy behaviors among youths, as early detection of such behaviors and their subsequent modifications can significantly improve every aspect of health and reduce the risk of chronic diseases later in life [31].

*The objective* of the study is to identify unhealthy behavior among university students; establish the means of detection of unhealthy behavior; identify the obstacles to volunteering; obtaining the relationship between volunteer preferred style of volunteering and the obstacles to volunteering.

The article "Healthcare Communication Role in the Detection of Unhealthy Behavior in University Students" was retracted in 2023. Reasons: signs of a paper mill; suspected computer-generated content; unreliable results or conclusions; concerns about the data.

## 2. Methods

In order to gather data for the study, an anonymous structured questionnaire was administered to both students and staff at Princess Nourah Bint Abdulrahman University, Riyadh, Saudi Arabia. 207 validly filled questionnaires were retrieved. The respondents were all females within the age range from 18 to more than 35 years.

The questionnaire for this study was developed by the authors (Table 1). It was in the Arabic language and had never been used before.

The data was collected by using the self-administered questionnaire (Table 1). It consists of two sections as follows.

Section 1 included sociodemographic characteristics and properties of participants such as age and gender—views on different facets of volunteering, unhealthy behaviors, and correlation between volunteering and unhealthy behaviors.

Section 2 consists of four axes. The first axis aims to explore the importance of volunteer work from the point of view of the volunteer. This part of the questionnaire contained 17 questions using a Likert scale of 5 points; totally agree = 5, agree = 4, neutral = 3, disagree = 2, and totally disagree = 1. Second axis: This axis aimed to measure the reasons for the existence of the phenomenon of offending behaviors on campus from the point of view of general volunteers. It was composed of 15 questions using a Likert scale of 5 points (totally agree = 5, agree = 4, neutral = 3, disagree = 2, and totally disagree = 1). The third axis focused on directing volunteer efforts of the students, professors, and human resources at the university for early detection of offending behavior in the university and establish a mechanism to reduce it. This part of the questionnaire contains 22 questions using a Likert scale totally agree = 5, agree = 4, neutral = 3, disagree = 2, and totally disagree = 1). The fourth axis aimed to elaborate reasons for participation and assistance mechanisms to detect the offending behavior in the university. This part of the questionnaire contains 16 questions using a Likert scale totally agree = 5, agree = 4, neutral = 3, disagree = 2, and totally disagree = 1). The questionnaire has been piloted to ensure face validity and has resolved both improvements in terminology and ease of use. However, the data collected from the pilot study were not involved in the final analysis. In terms of reliability, a variety of factors have been taken into account when planning this analysis to reduce the risk to reliability. The data gathered was subjected to Statistical Package for Social Science (SPSS) 2020. Descriptive statistics were used to report the percentages for definite variables, while mean values with standard deviations were used to report continuous variables. Missing data were omitted on the basis of analysis-by-analysis and valid percentages were reported. The data was also subjected to correlation analysis to determine the relationship between the volunteer preferred style of volunteering and the obstacles to volunteering.

The article "Healthcare Communication Role in the Detection of Unhealthy Behavior in University Students" was retracted in 2023. Reasons: signs of a paper mill; suspected computer-generated content; unreliable results or conclusions; concerns about the data.

## 3. Results

The demographic characteristics of the respondents revealed ages ranging from 18 years to above 35 years. It is not surprising that the marital status of most (92.8%) of the respondents was single as the sample population comprised mainly students (Table 2.

Regarding the source of income of the respondents, most (42%) of the respondents had their source of income from university rewards; this is followed by 25.1% of the respondents whose source of personal income was from all of the university rewards, parents, and grandparents. Others had their personal source of income ranging from monthly salary, husband, internship, donation and alms, business, social security, charities, and other sources as listed in Table 3.

With regard to the mode of volunteering, it seems that online life affected the expected voluntary behaviors. Results showed that 30% of the respondents prefer to volunteer through groups. This percentage was expected to be more, but it was less due to the online life period since students cannot meet and work in groups. The results also show that most of the respondents nowadays prefer electronic volunteering due to the limitation of gathering and outdoor activities (Table 4).

Lack of time constitutes the greatest obstacle to digital volunteering, representing almost half (48.8%) of the entire data, while lack of conviction/interest/time constitutes the least obstacle (0.5%). Other factors that hinder digital volunteering, as shown by the table, include lack of time + weak interest (15.0%), lack of awareness, and culture (7.2%) (Table 5).

University administration has a positive role in the development of volunteering work. It is also observed that volunteering positively affects university volunteers. This is seen as most of the respondents agreed that volunteering enabled them to develop enough interest to strive to continually update their information as development in the field persists. Most respondents reported enhanced communication skills; other positive roles include improved ability to tackle problems and development of basic skills in the use of technology, as shown in Table 6.

From Table 7, only 28 (13.5%) of the 207 respondents reported using social media in detecting women with offending behavior.

When considering the most widely used methods of communication, Twitter is the most widely used method of communication as 50% (14) of the respondents (28) make use of it. This was followed by both Twitter and Instagram and Twitter, Snapchat, Phone calls, YouTube, LinkedIn, WhatsApp, and Telegram, which were utilized by 3 (1.4%) of the respondents each. 2 (1%) of the respondents use Snapchat as a medium of communication, another 2 (%) of them utilize Twitter coupled with surfing the web; 1 (0.5%) of the respondents browse the web only as a means of communication (Table 8 and Figure 1.

The article "Healthcare Communication Role in the Detection of Unhealthy Behavior in University Students" was retracted in 2023. Reasons: signs of a paper mill; suspected computer-generated content; unreliable results or conclusions; concerns about the data.

Table 9 shows the mean and standard deviation of reasons for participation and assistance mechanism to detect unhealthy behavior in the university.

Table 10 shows that 37 (17.9%) of the respondents indicated that Attack on Others and Properties is the most prevalent unhealthy behavior found among university students; this is followed by bullying/insults/verbal abuse and bullying (13.5%) and (8.7%), respectively.

Most of the respondents (70) who do volunteer work do it in the Princess Nourah University and have revealed to have helped detect unhealthy behavior among women. Others carry out their volunteering work at Community development association (11), charitable association (5), outside the university (10), and both within and outside the university (21); the only respondent who carries out volunteer work electronically has not helped to detect any kind of unhealthy behavior (Table 11).

As shown in Table 12, the value of Pearson's R is 0.245; thus, it is considered a weak or no correlation. There is hence no correlation between how respondents preferred volunteer work and the obstacle to volunteering. There is not much difference in the obstacles to volunteering faced by respondents despite their preferred style of volunteering.

With regard to the correlation between the four themes/axes of this study, we have the following. The first axis: the importance of volunteer work from the point of view of the volunteer; the second axis: the reasons for the existence of the phenomenon of offending behaviors on campus from the point of view generally volunteers; third *axis*: directing Volunteer efforts of the students, professors and human resources at the university for early detection of offending behavior in the university and establish a mechanism to reduce it; the fourth axis: reasons for participation and assistance mechanism to detect the offending behavior in the university by those who actually participated.

From Table 13, the correlation between the first and second axis is 0.139 indicating a weak relationship between the importance of volunteer work from the point of view of the volunteer and the reasons for the existence of the phenomenon of offending behaviors on campus from the point of view generally volunteers. The Sig. (2-tailed) is 0.045, indicating that there is no statistically significant correlation between the two variables. The correlation between the first and third axis and the first and fourth axis is 0.431 and 0.369, respectively, also indicating that there is no correlation between each pair of variables. Of all the variable pairs represented in the above table, there is only a moderate correlation between the third and fourth axis, thus indicating that there is a relationship between the two variables.

The article "Healthcare Communication Role in the Detection of Unhealthy Behavior in University Students" was retracted in 2023. Reasons: signs of a paper mill; suspected computer-generated content; unreliable results or conclusions; concerns about the data.

## 4. Discussion

This study was of clearly stated objectives. The features of the respondents were well represented; randomized sampling was also utilized; since the sample profile is composed of students, this enables easy access and low cost for data collection. On the other hand, a limited number of previous studies related to this topic was reported.

As comparing this study with other previously reported studies, the results of this study showed that youth and young adults form a greater part of volunteering. This is not surprising as the *Arab News* reported that “the majority of Saudi youth would be more than willing to get involved in volunteer work, according to a survey” [32]. Volunteer work span across all work ages, university education level, occupation, and marital status. It is revealed that most volunteers prefer volunteering in groups.

Contrary to Sills' classic study on volunteering [33], people not only engage in volunteer work for altruistic motives only but also for other beneficial rewards such as learning new skills and self-development among others [34]. A major obstacle to volunteering is the lack of time (48.8%). Of the unhealthy behavior revealed in this study, attacks on others and properties were the most frequent (17.9%). This was followed by bullying, insults, and verbal abuse (13.5%). Bullying is obviously among the top list of unhealthy behavior as it takes several forms [35, 36], from cyber-bullying to face-to-face bullying, insults, and verbal abuses.

On a global scale, there is rising anticipation that volunteers will cover a bigger responsibility in disaster management and disaster risk diminution in time to come than it has in the past. This is propelled by an increasing global focus on creating “resilience to disasters through a “bottom-up” process in the form of volunteer initiatives rooted in the community” [19]. Lately, this focus was reemphasized in the 2015–2030 Sendai agenda for Disaster Risk Reduction, arrogated by the United Nation's March 2015 General Assembly [37]. The guideline demanded that “responsibilities be shared” covering all stakeholders and sectors of society and vociferates “an all-of-society engagement and partnership.” Also, it renders an extensive catalog of proceedings for “civil society, volunteers, organized voluntary work organizations and community-based organizations” that states should encourage.

The article "Healthcare Communication Role in the Detection of Unhealthy Behavior in University Students" was retracted in 2023. Reasons: signs of a paper mill; suspected computer-generated content; unreliable results or conclusions; concerns about the data.

Nevertheless, the outlook of volunteering is gradually shifting in the twenty-first century in manners that bring significant problems and chances for disaster management. Particularly, shifts in the pattern of paid jobs, values, and lifestyles, and the latest technology has resulted in a reduction in “traditional,” time-consuming, high dedication volunteering and an increase in more vast, flexible and periodic patterns of volunteering [38]. Considerably, “volunteer strategies in the emergency management sector still depend profoundly on the customary model of volunteering” [39, 40].

Volunteering definitions are changing, alongside the act of volunteering [41, 42]. In Australia, the highest national body lately arrogated a more comprehensive definition: “Volunteering is time willingly given for the common good and without financial gain” [43, 44]. The recent definition cuts across a greatly wider array of budding and less conventional kinds of volunteering juxtaposed to the past, including unofficial and periodic volunteering, group volunteering where a member of staff time is contributed, electronic or online volunteering, and activism. This kind of shift towards more general knowledge of what makes up volunteering in the contemporary perspective is accompanied by the likelihood of higher acknowledgment, legitimacy, and protection for the greater variety of volunteering that has constantly taken place in disaster situations. However, greater recognition also brings the prospective for more government mediation, which stressed has tendency to influence the drives and developing behaviors that inspire unofficial volunteering negatively [42]. Results of the study were manifested earlier in a Research Square, preprint document [45], showing that the majority of Saudi youth are more willing to be involved in volunteer work.

## 5. Conclusions

The findings reveal that digital volunteering is effectively gaining ground in the detection and management of unhealthy behaviors among university students. Much more could be achieved through digital volunteering if more awareness is created and volunteering programs are designed to be more interesting and less time-consuming to allow more students to participate. Based on these facts, this study hereby makes the following recommendations: more opportunities should be given to students to participate in volunteering work. There should be proper awareness and orientation about new and existing volunteering work. Students should be encouraged to participate in digital volunteering. Students should be afforded opportunities to volunteer outside the university and access the diversity of volunteer opportunities. There should be partnerships among the university, institutions, and volunteer associations, which will give another character to female students and develop extracurricular thinking skills for female volunteers, as there are specializations that pay more attention to this aspect, as is the case in the disciplines of social service, psychology and others. Volunteer programs should be designed to be less time-consuming and more interesting to students while serving the purpose for which there were created.

The article "Healthcare Communication Role in the Detection of Unhealthy Behavior in University Students" was retracted in 2023. Reasons: signs of a paper mill; suspected computer-generated content; unreliable results or conclusions; concerns about the data.

## Figures and Tables

**Figure 1:** Most widely used methods of communication.

**Table 1:** Self-administered questionnaire to identify unhealthy behaviors among university students and directing volunteering to establish means of detection and minimization of unhealthy behavior.

Variable		Description
The first axis: the importance of volunteer work from the point of view of the volunteer		
1	Interested in the field of voluntary work of any kind	
2	Academic specialization is important in the field of voluntary work	
3	Interested in volunteering subject	
4	Age is important in the field of voluntary work	
5	I am aware of the concept and importance of voluntary work	
6	University administration has a positive role in the development and supervision of voluntary work and supervision	
7	I had the opportunity to practice voluntary work on campus	
8	I am aware of the procedures used to carry out volunteer work on campus	
9	There is follow-up and monitoring of volunteer work on campus	
10	I have participated in several voluntary activities in the campus	
11	I feel good in general about the level of organization of volunteer work on campus	
12	Volunteer work had improved my communication skills	
13	Voluntary work had helped me in development of interest in improving my continuous update of my knowledge in the field	
14	Volunteer work improved my ability to investigate and solve new problems	
15	Volunteer work developed my ability to work effectively with groups	
16	Volunteer work helped me to develop basic skills in the use of technology	
17	Burden of study negatively affect the voluntary work	
The second axis: the reasons for the existence of the phenomenon of offending behaviors on campus from the point of view generally volunteers		
18	The lack of monitoring on campus facilitated unhealthy behavior	
19	Lack of home control, education, and proper values facilitated unhealthy behavior	
20	Careless attitude of parents and consider it normal behavior	
21	The university officials ignorance towards abnormal behavior and considering it accepted	
22	Lack of awareness and mechanisms for early detection of offending behavior in the university	
23	The absence of syllabus or courses	
24	The availability of free time for the student due to few credit hours	
25	To keep up with the largest number of rich friends because the behavior is promoted and have the freedom and civilization	
26	The lack of strict sanctions and regulations of the organization live up to the offending behavior	
27	Non-implementation of sanctions issued and applied without sufficient application	
28	Not transfer erring behaviorally to the judiciary or the law, and sufficing with internal punishment	
29	Secrecy and opacity on the subject and not to reveal the offending behavior of the specialists or all	
30	Means of communication and docility behind their websites and advertisements facilitate the imitate the offending behavior and its implementation	
31	Lack of awareness of the impact of the offending behavior has done later and the difficulty of their involvement in society and the difficulty of job opportunities	
32	The lives of luxury, extravagance and wealth for some students, which they want to show to their peers	
Third axis: directing volunteer efforts of the students, professors and human resources at the university for early detection of offending behavior in the university and establish a mechanism to reduce it		
33	Activities and community service in the college are interested in volunteering and direction to reduce offending behavior	
34	There are suitable training opportunities for the development of voluntary work to reduce offending behavior on campus	
35	I have learned the volunteer tasks assigned to me in the field of reducing offending behavior	
36	You have the volunteer skills necessary to perform the tasks assigned to you to reduce offending behavior	
37	I feel good about myself if involved in reducing offending behavior	
38	Volunteer work to reduce the offending behavior has a positive role in the university community	
39	What I have learned in volunteer work to reduce offending behavior will be important for the future	
40	I have problems while volunteering on campus, especially to reduce offending behavior	
41	The campus volunteer work hours suit me in reducing offending behavior	
42	Ready to train in nora tender volunteer incubator inside the campus is working to reduce offending behavior	
43	Holds a national voluntary work permit	
44	I follow nora tender volunteer platform that offers volunteer opportunities	
45	My hours for volunteer work are counted in the skill register	
46	There are clear announcements and instructions at the university of volunteer work to reduce offending behavior	
47	I joined the forums and workshops held by the university to spread the culture of volunteer work to reduce offending behavior	
48	I am informed by the responsible authorities of the dates of volunteer work to reduce offending behavior in accordance with the statutory procedures	
49	I am aware of the goals and motivations and mechanisms of volunteering to reduce offending behavior	
50	I am aware of the most important volunteer fields and forms to reduce offending behavior	
51	I have to know how to attract volunteers to reduce offending behavior	
52	Faculty members cooperate with me to facilitate voluntary work tasks to reduce offending behavior	
53	Volunteer work to reduce offending behavior finds solutions to community problems	
54	Volunteer work to reduce offending behavior finds solutions to community problems	
The fourth axis: reasons for participation and assistance mechanism to detect the offending behavior in the university ∗ those who actually participated		
55	The person who carried out the offending behavior contacted strangers through social networks to help her in the implementation of the offending behavior and I discovered that	
56	People on and off campus helped me uncover who did the offending behavior and the methods she used to commit the offending behavior	
57	I imitated what is shown on social networks to contribute to the detection of offending behavior	
58	I asked for help from colleagues, specialists and security guards in order for me to participate in the detection of the offending behavior	
59	I learned through courses, workshops, cultural clubs and extracurricular activities about the types of offending behavior and how to monitor it	
60	My exposure to blackmail by those who do the offending behavior and my rejection of the behavior prompted me to participate in monitoring the offending behavior.	
61	My ability to hack the websites and influencing others helped me to monitor the offending behavior	
62	Advertisement and invitations in the university led me to participate in reducing offending behavior	
63	My friends volunteer in reducing offending behavior, encouraging me with their experiences, to experiment with monitoring the offending behavior	
64	My values and principles of religion made me motivated to participate in the monitoring of the offending behavior for the satisfaction of God	
65	My knowledge of the types of offending behavior and harm to the individual and society encouraged me to fight	
66	Peer indifference to the matter, out of fear, irresponsibility, or distance from problems, was frustrating me on the one hand and encouraging me, on the other hand, to uncover the offending behavior and follow-up and continue doing so	
67	My ability to hide my true character on campus easy to expose students who committed offending behavior	
68	My desire to do good and feeling safe on campus motivated me to participate and take initiative	
69	My sense of security in terms of ease of tracking and lack of regulatory laws made it easy for me to contribute to uncovering the offending behavior	
70	Guidance and counseling by professors, clubs, volunteers and the community service agency raised my spirits, so I made the offending behavior and detection of it my priority	

The article "Healthcare Communication Role in the Detection of Unhealthy Behavior in University Students" was retracted in 2023. Reasons: signs of a paper mill; suspected computer-generated content; unreliable results or conclusions; concerns about the data.

**Table 2:** Sociodemographic characteristics of the respondents.

Variable	Frequency	Percent
Age		
18 to 23 yrs	169	81.6
24 to 28 yrs	31	15.0
29 to 34 yrs	2	1.0
35 yrs and above	5	2.4
Total	207	100.0

University education level		
1st year	4	1.9
2nd year	54	26.1
3rd year	14	6.8
4th year	16	7.7
After 5th year	109	52.7
Postgraduate	10	4.8
Total	207	100.0

Marital status		
Single	192	92.8
Married	14	6.8
Divorced	1	.5
Total	207	100.0

Occupation		
Student	178	86.0
Student + self-employed	6	2.9
Self-employed	4	1.9
Partly employee	19	9.2
Total	207	100.0

Monthly income of the family		
Less than SR 3,000	36	17.4
3,000 to 3,499 riyals	22	10.6
3,500 to 4,900 riyals	11	5.3
5,000 to 6,499 riyals	4	1.9
6,500 to 7,999 riyals	6	2.9
8,000 to 10,000 riyals	19	9.2
Above 10,000 riyals	67	32.4
Undefined/unspecified	42	20.3

Total	207	100.0

**Table 3:** Source of personal income of respondents.

Source of personal income	Frequency	Percent
No job	1	0.5
University reward	87	42.0
University reward/parents/grandparents	52	25.1
Parents/grandparents	12	5.8
Donation and alms	1	0.5
Monthly salary	2	1.0
Position after the university	18	8.7
Position after the university/university	12	5.8
Reward/parents/grandparents		
Husband	6	2.9
University reward/parents/grandparents/social security	2	1.0
Position after the university/university	2	1.0
Reward/charity/social security		
Internship	6	2.9
University/social security	2	1.0
Position after the university/university	1	0.5
Reward/husband		
Position after the university/husband	1	0.5
University reward/business	1	0.5
Position after the university/charity/social security	1	0.5

Total	207	100.0

**Table 4:** How do you prefer volunteering?

Variable	Frequency	Percent
In group	63	30.4
Individual	10	4.8
Group (in hospital)	37	17.9
Individual/group	10	4.8
Individual/group/electronic	21	10.1
Individual/group/electronic/cafe/coffee shop	39	18.8
Individual/group/hospital	16	7.7
Group/electronic	9	4.3
Individual/electronic	2	1.0
Total	207	100.0

The article "Healthcare Communication Role in the Detection of Unhealthy Behavior in University Students" was retracted in 2023. Reasons: signs of a paper mill; suspected computer-generated content; unreliable results or conclusions; concerns about the data.

**Table 5:** Obstacles to volunteering.

Obstacles to volunteering (variables)	Frequency	Percent	Cumulative percent
Lack of time	101	48.8	48.8
Lack of awareness and culture	15	7.2	56.0
Lack of interest	11	5.3	61.4
Lack of time + weak interest	31	15.0	76.3
Lack of time + lack of conviction	8	3.9	80.2
Lack of time/conviction/awareness	16	7.7	87.9
Lack of conviction/interest/time/awareness	4	1.9	89.9
Lack of time/conviction/awareness/culture/interest	11	5.3	95.2
Lack of conviction	3	1.4	96.6
Lack of conviction/interest/time	1	0.5	97.1
Lack of awareness/culture/Interest	3	1.4	98.6
Lack of time and transport	3	1.4	100.0
Total	207	100.0	

**Table 6:** Effect of volunteering on university volunteers.

Variable	Frequency	Percentage
University administration has a positive role in the development of volunteering work		
Strongly agree	80	38.6
Agree	84	40.6
Neutral	38	18.4
Disagree	3	1.4
Strongly disagree	2	1.0
Total	207	100.0

Volunteering triggered me to update my information as development in the field		
Strongly agree	71	34.3
Agree	78	37.7
Neutral	36	17.4
Disagree	16	7.7
Strongly disagree	6	2.9
Total	207	100.0

Volunteer work improved my ability to investigate and solve problems		
Strongly agree	61	29.5
Agree	65	31.4
Neutral	44	21.3
Disagree	29	14.0
Strongly disagree	8	3.9
Total	207	100.0

Volunteer work improved my communication skills		
Strongly agree	87	42.0
Agree	74	35.7
Neutral	41	19.8
Disagree	5	2.4
Strongly disagree	0	0
Total	207	100.0

Volunteer work helped me develop basic skills in the use of technology		
Strongly agree	67	32.4
Agree	84	40.6
Neutral	44	21.3
Disagree	9	4.3
Strongly disagree	3	1.4

Total	207	100.0

**Table 7:** Social media in detecting women with unhealthy behavior.

		Frequency	Percent	Valid percent	Cumulative percent
Valid	Yes	28	13.5	13.5	13.5
	No	179	86.5	86.5	100.0
	Total	207	100.0	100.0	

**Table 8:** The most widely used method of communication.

How do you prefer volunteering?	The most widely used method of communication								
	Snapchat	Twitter	Snapchat/Twitter	Twitter/Snapchat/Instagram	Twitter/Snapchat/Phone Calls/Youtube/LinkedIn/WhatsApp/Telegram	Twitter and Instagram	Browse the web	Twitter/browse the web	Total
In group	0	10	1	0	0	0	0	2	13
Individual	0	0	0	0	1	0	0	0	1
Group (in hospital)	0	1	0	1	0	1	0	0	3
Individual/group	0	0	1	0	0	0	0	0	1
Individual/group/electronic/h	2	0	0	0	0	2	1	0	5
Individual/group/electronic/cafe/coffee shop	0	3	0	0	2	0	0	0	5
Total	2	14	2	1	3	3	1	2	28

**Table 9:** Reasons for participation and assistance mechanism to detect the unhealthy behavior in the university.

		CK	CL	CM	CN	CO	CP	CR	CT	CU
N	*Valid*	164	163	162	163	164	163	163	162	163
	*Missing*	43	44	45	44	43	44	44	45	44
Mean		2.9329	3.0000	2.7531	2.8650	2.4695	2.5153	2.7853	2.4198	2.5276
Std. deviation		1.24896	1.20185	1.08096	1.12500	.99338	1.07356	1.08720	1.01375	1.05592

CK = my exposure to blackmail by those who do the unhealthy behavior and my rejection of the behavior prompted me to participate in monitoring the offending behavior. CL = my ability to hack the websites and influencing others helped me to monitor unhealthy behavior. CM = advertisement and invitations in the university led me to participate in reducing unhealthy behavior. CN = my friends volunteer in reducing unhealthy behavior, encouraging me with their experiences, to experiment with monitoring the unhealthy behavior. CO = my values and principles of religion made me motivated to participate in the monitoring of unhealthy behavior for the satisfaction of God. CP = my knowledge of the types of offending behavior and harm to the individual and society encouraged me to fight. CR = peer indifference to the matter, out of fear, irresponsibility, or distance from problems, was frustrating me on the one hand and encouraging me, on the other hand, to uncover unhealthy behavior and follow-up and continue doing so. CT = gy sense of security in terms of ease of tracking and lack of regulatory laws made it easy for me to contribute to uncovering the offending behavior. CU = guidance and counseling by professors, clubs, volunteers, and the Community Service Agency raised my spirits, so I made the unhealthy behavior and detection of it my priority.

The article "Healthcare Communication Role in the Detection of Unhealthy Behavior in University Students" was retracted in 2023. Reasons: signs of a paper mill; suspected computer-generated content; unreliable results or conclusions; concerns about the data.

**Table 10:** Unhealthy behavior detected by respondents.

Unhealthy behaviors		Frequency	Percent
Valid	Smoking/drug abuse	7	3.4
	Sexual abnormalities	2	1.0
	Bullying/insults/verbal abuse	28	13.5
	Theft	6	2.9
	Attack on others and properties	37	17.9
	Bullying	18	8.7
	Smoking and bullying	2	1.0
	Sexual abnormalities and bullying	1	0.5
	Sexual abnormalities/extortion/bullying/insults/verbal abuse	4	1.9
	Inappropriate disposal of waste/refuse	1	0.5
	Drug abuse/wrong use of medication	1	00.5
	Total	107	51.7
Missing	System	100	48.3
Total		207	100.0

**Table 11:** Detection of unhealthy behavior.

		Have you ever helped to detect any kind of unhealthy behavior?			Total
		Did not reveal	Yes	No	
Where do you do your volunteer work?	None	2	31	24	57
	Princess Nourah University/Hospital/Ministry of Health	1	31	38	70
	Community development association	0	11	3	14
	Charitable association	0	5	8	13
	Outside the university	0	10	5	15
	Both within and outside the university	1	21	15	37
	Electronically	0	0	1	1
Total		4	109	94	207

**Table 12:** Correlation between how respondents prefer volunteer work and the obstacle to volunteering.

		Symmetric measures			
		Value	Asymp. std. error^a^	Approx. T^b^	Approx. sig.
Interval by interval	Pearson's R	0.245	0.057	3.624	0.000^c^
Ordinal by ordinal	Spearman correlation	0.231	0.064	3.405	0.001^c^
N of valid cases		207			

^a^Not assuming the null hypothesis. ^b^Using the asymptotic standard error assuming the null hypothesis. ^c^Based on normal approximation.

The article "Healthcare Communication Role in the Detection of Unhealthy Behavior in University Students" was retracted in 2023. Reasons: signs of a paper mill; suspected computer-generated content; unreliable results or conclusions; concerns about the data.

**Table 13:** Correlation between the four themes/axes of this study.

		Correlations			
		First axis	Second axis	Third axis	Fourth axis
First axis	Pearson correlation	1	0.139^∗^	0.431^∗∗^	0.369^∗∗^
	Sig. (2-tailed)		0.045	0.000	0.000
	N	207	207	207	168

Second axis	Pearson correlation	0.139^∗^	1	0.279^∗∗^	0.258^∗∗^
	Sig. (2-tailed)	0.045		0.000	0.001
	N	207	207	207	168

Third axis	Pearson correlation	0.431^∗∗^	0.279^∗∗^	1	0.665^∗∗^
	Sig. (2-tailed)	0.000	0.000		0.000
	N	207	207	207	168

Fourth axis	Pearson correlation	0.369^∗∗^	0.258^∗∗^	0.665^∗∗^	1
	Sig. (2-tailed)	0.000	0.001	0.000	
	N	168	168	168	168

^∗^Correlation is significant at the 0.05 level (2-tailed). ^∗∗^Correlation is significant at the 0.01 level (2-tailed).

## Data Availability

Any raw data or materials used in the preparation of this manuscript are available upon reasonable request to Dr. Samar Alshawwa (szalshawwa@pnu.edu.sa).
